The article "Meta-analysis of the associations between TNF-α or IL-6 gene polymorphisms and susceptibility to lung cancer" was retracted in 2016. Reasons: compromised peer review; concerns about the authorship; concerns about a third party's involvement.

# Meta-analysis of the associations between TNF-α or IL-6 gene polymorphisms and susceptibility to lung cancer

**DOI:** 10.1186/s40001-015-0113-9

**Published:** 2015-03-21

**Authors:** Wei Zhou, Shuxiang Zhang, Yingchun Hu, Jianrong Na, Na Wang, Xuan Ma, Lizhi Yuan, Fanzhen Meng

**Affiliations:** Department of Respiration, General Hospital of Ningxia Medical University, Shengli Street, Yinchuan, 750004 China

**Keywords:** Lung cancer, Tumor necrosis factor-alpha, Interleukin 6, Gene polymorphisms, Meta-analysis

## Abstract

**Background:**

Several studies have indicated an association between tumor necrosis factor-alpha (TNF-α) or interleukin (IL)-6 gene polymorphisms and lung cancer risk. However, the conclusions remain controversial.

**Methods:**

An English literature screening about case-control trials with regard to TNF-α (-308G/A) or IL-6 (174G/C) polymorphisms and lung cancer susceptibility was performed on PubMed, EMBASE, and EBSCO until November 2012. The pooled odds ratio (OR) and 95% confidence intervals (CI) were calculated using STATA 11.0. Sensitivity analysis was performed by sequential omission of individual studies. Publication bias was evaluated by Egger’s linear regression test and funnel plots.

**Results:**

Eight eligible studies, including 1,690 patients and 1,974 controls, were identified in this meta-analysis. Compared with the control, no significant association was revealed between TNF-α-308G/A (GG + GC vs. CC: OR = 1.10, 95% CI: 0.73 to 1.64; GG vs. GC + CC: OR = 1.02, 95% CI: 0.81 to 1.27; GC vs. CC: OR = 1.13, 95% CI: 0.73 to 1.77; GG vs. CC: OR = 1.04, 95% CI: 0.80 to 1.36; G vs. C: OR = 1.03, 95% CI: 0.90 to 1.18) or IL-6 174G/C (GG + GC vs. CC: OR = 1.10, 95% CI: 0.73 to 1.64; GG vs. GC + CC: OR = 1.02, 95% CI: 0.81 to 1.27; GC vs. CC: OR = 1.13, 95% CI: 0.73 to 1.77; GG vs. CC: OR = 1.04, 95% CI: 0.80 to 1.36; G vs. C: OR = 1.03, 95% CI: 0.90 to 1.18) and lung cancer risk. The pooled OR remained unchanged after removing the maximum-weight study and no publication bias was observed.

**Conclusions:**

The study raises the possibility of no correlation between the polymorphisms of the two genes and lung cancer susceptibility. However, further researches with large-sample or subgroup analyses are necessary to validate the conclusions.

## Background

Lung cancer is one of the most common causes of cancer-related mortality worldwide, being responsible for approximately 87,750 deaths in men and 72,590 in women in 2012 [1]. Although air pollution and smoking are believed to be important contributory factors for the development of lung cancer [2], only one in ten persons exposed to air pollution or tobacco ultimately develops lung cancer, indicating that other factors, like genetic factors, are also important as well [3].

Recently, growing evidence suggest that chronic inflammation may exert important roles in the etiology of lung cancer [4]. Cytokines from inflammatory cells can increase intracellular reactive oxygen and nitrogen species and cause DNA damage and epigenetic changes (that is, promoter hyper-methylation), eventually silencing tumor suppressors and promoting tumor initiation [4]. Regulation of pro-inflammatory cytokine expressions can inhibit tumor cell proliferation, angiogenesis, invasion, and meta-stasis, but stimulate cells apoptosis [5,6].

Tumor necrosis factor-alpha (TNF-α) and interleukin (IL)-6 are pleiotropic cytokines involved in inflammatory response and cancer pathogenesis. Previous studies have indicated that the high levels of both cytokines are directly correlated with the short survival of lung cancer patients [7,8]. It is well known that genetic variants, especially the functional polymorphisms located in the promoter region of candidate genes, may quantitatively change the gene’s expression [9]. Therefore, several studies have been performed to investigate the associations between the polymorphisms of the TNF-α (-308G/A) or IL-6 (174G/C) and susceptibility to lung cancer. However, the conclusions remain controversial. Shih *et al*. demonstrated that the patients carrying a homologous AA or heterologous GA genotype at TNF-α-308 had a tendency to develop into advanced disease [10]. Colakogullari *et al*. reported that the IL-6 (174G/C) heterozygous genotype occurred at a higher frequency in lung cancer patients while the homozygous form (G/G) was more common in healthy controls [11]. No associations were seen between TNF-α or IL-6 polymorphisms and the risk of lung cancer by Seifart *et al*. [12]. These inconsistent conclusions may result from the small-sample size in each study and different inclusion criteria as well as other factors. Therefore, it is essential to carry out a meta-analysis to quantitatively integrate the results of previous reports and comprehensively evaluate their association, which was not reported.

## Methods

### Literature screening

Eligible studies were identified by searching electronic databases including PubMed (http://www.ncbi.nlm.nih.gov/pubmed/), Excerpt Medica Database (EMBASE, http://www.elsevier.com/online-tools/embase), and EBSCOhost Online Research Databases (EBSCO, http://www.ebscohost.com/) for relevant reports published before November 2012 using the following terms: (TNF OR tumor necrosis factor OR IL-6 OR interleukin 6) AND (Lung Cancer OR lung carcinoma OR lung tumor) AND (polymorphism OR polymorphisms OR variant OR variants). The computer search was supplemented with manual searches for reference lists of all retrieved review articles, primary studies, and abstracts from meetings to retrieve additional studies.

### Inclusion and exclusion criteria

The following criteria were used to enroll studies published in English: (1) case-control trials with raw data published before November 2012, without the limitation of the research time, (2) the study investigates the associations between TNF-α-308G/A or IL-6-174G/C and lung cancer susceptibility, and (3) the size of the samples, distribution of alleles, genotype frequency, or other information are available for both cases and controls.

Studies were excluded if one of the following existed: (1) the design was based on family or sibling pairs, (2) data were collected from the overview or summary, (3) the literatures were duplicate publications, and (4) there was insufficient information for data extraction.

### Data extraction

Two system evaluators independently searched and screened the literatures. Data extraction was performed in accordance with a pre-set form while inconsistencies in the process were discussed or referred to a third party. The following data were extracted: first author, publication date, original research site, race, age of case, number of case, number of control, type of control, the polymerase chain reaction (PCR) method used for genotyping, and whether the gene distribution of the controls was in compliance with the Hardy-Weinberg Equilibrium (HWE).

### Statistical analysis

The pooled odds ratio (OR) and 95% confidence intervals (CI) were calculated as the integrative indicators to assess the associations between TNF-α-308G/A or IL-6-174G/C and lung cancer susceptibility. Chi-square-test-based *Q* statistic and *I*^*2*^ were used as the heterogeneity indicators. If the result of the *Q* test was *P*_Q_ < 0.05 or *I*^2^ ≥ 50%, indicating the presence of heterogeneity, a random-effects model was used to estimate the OR. Otherwise, a fixed-effects model was used. For each polymorphic locus, five comparison models, including dominant model, recessive model, heterozygous genotype comparison, homozygous genotype comparison, and allele comparison, were carried out. We checked the genotype distribution of the controls if the papers did not describe it.

To explore the heterogeneity across studies for the dominant model of TNF-α-308G/A and lung cancer susceptibility, subgroup analyses according to region distribution and detection method and meta-regression were performed. Sensitivity analysis was performed by sequential omission of individual studies. Publication bias was evaluated by Egger’s linear regression test [13]. Finally, publication bias was explored by Egger’s linear regression test and funnel plots.

All statistical analyses were conducted by STATA 11.0 (Stata Corporation, College Station, TX, USA). All the *P* values were determined from two-sided test and the significant level was set at 0.05.

## Results

### Literature search and screening results

A total of 196 literatures were retrieved and screened through reading title and abstract to remove duplicate, non-case-control and non-target studies. Review of the full text of the 13 articles further excluded five articles: three did not study TNF-α-308G/A or IL-6-174G/C and two did not include allele frequency data. As a result, a total of eight relevant studies [10-12,14-18] were included in this meta-analysis, among which six studies were [10-12,14-16] about TNF-α-308G/A and four studies about IL-6-174G/C [11,12,17,18] (Figure 1).

**Figure 1:** **Flow chart for literature screening.**

### Basic information of the included studies

Tables 1 and 2 show the main features of the included studies and genotype distribution, respectively. Seven out of the eight studies were carried out in Europe while only one in Asia. These studies were published during 2004 to 2010. Most of the controls consisted of healthy people, matching with the cases in age, sex, place of residence, occupation, and other factors. There was no study with genotype distribution departing from HWE.

**Table 1:** **Basic information for studies included**

**First author**	**Year**	**Country**	**Ethnicity**	**Polymorphisms**	**Number of cases**	**Number of controls**	**Method**	**HWE**
Helmig	2010	Germany	European	TNF-α 308G/A	374	177	Real-time PCR	Yes
Flego	2009	Croatia	European	TNF-α 308G/A	230	230	PCR-RFLP	Yes
Stankovic	2009	Serbia	European	TNF-α 308G/A	70	102	PCR-RFLP	Yes
Colakogullari	2008	Turkey	European	TNF-α 308G/A IL-6 174G/C	44	59	PCR-SSP	Yes
Vogel	2008	Denmark	European	IL-6 174G/C	403	744	PCR	Yes
Seifart	2006	Germany	European	TNF-α 308G/A IL-6 174G/C	117	243	PCR-RFLP	Yes
Shih	2006	China	Asian	TNF-α 308G/A	202	205	PCR-RFLP	Yes
Campa	2004	Norway	European	IL-6 174G/C	250	214	Taqman	Yes

TNF: tumor necrosis factor; IL: interleukin; PCR: polymerase chain reaction; PCR-RFLP: polymerase chain reaction-restriction fragment length polymorphism; PCR-SSP: polymerase chain reaction-sequence specific primer; HWE: Hardy-Weinberg Equilibrium.

**Table 2:** **Distribution of genotype and allele for TNF-α-308G/A and IL-6-174G/C**

**Locus**	**Research**	**Number of case**			**Number of control**			**Number of case**		**Number of control**	
		**GG**	**GA**	**AA**	**GG**	**GA**	**AA**	**G**	**A**	**G**	**A**
TNF-α 308G/A	Helmig *et al*.	290	79	5	136	38	3	659	89	310	44
	Flego *et al*.	169	52	9	171	53	6	390	70	395	65
	Stankovic *et al*.	57	13	0	71	28	3	127	13	170	34
	Colakogullari *et al*.	38	5	0	37	16	6	81	5	90	28
	Seifart *et al*.	29	11	0	171	67	4	69	11	409	75
	Shih *et al*.	110	75	15	169	34	2	295	105	372	38
		GG	GC	CC	GG	GC	CC	G	C	G	C
IL-6 174G/C	Colakogullari *et al*.	10	29	5	27	22	9	49	39	76	40
	Vogel *et al*.	105	202	96	204	361	179	412	394	769	719
	Seifart *et al*.	19	16	4	90	107	46	54	24	287	199
	Campa *et al*.	64	111	68	55	105	47	239	247	215	199

TNF: tumor necrosis factor; IL: interleukin.

### Combination of quantitative data

#### TNF-α-308G/A and lung cancer susceptibility

Six case-control studies investigated the association between the TNF-α-308G/A and lung cancer susceptibility, including 957 cases and 1,015 controls. The meta-analysis suggests that the TNF-α-308G/A polymorphism is not significantly associated with lung cancer risk in all the five comparison models with high heterogeneity (*I*^2^ > 50%) except GA vs. AA (dominant model, GG + GA vs. AA: OR = 0.95, 95% CI: 0.30 to 2.99, *P* = 0.935; recessive model, GG vs. GA + AA: OR = 1.07, 95% CI: 0.55 to 2.10, *P* = 0.834; heterozygous genotype comparison, GA vs. AA: OR = 0.81, 95% CI: 0.43 to 1.54, *P* = 0.524; homozygous genotype comparison, GG vs. AA: OR = 1.00, 95% CI: 0.27 to 3.62, *P* = 0.994; allele comparison, G vs. A: OR = 1.12, 95% CI: 0.58 to 2.14, *P* = 0.734) (Table 3). Forest plot for the dominant model of TNF-α-308G/A is shown in Figure 2.

**Table 3:** **Results for different comparison models**

**Locus**	**Comparison**	**OR (95% CI)**	***Z***	***P***_**A**_	***I*** ^***2***^	***P***_**Q**_	**Model**	**Egger’s test**	
								***t*** **value**	***P*** **value**
TNF-α 308G/A	GG + GA vs. AA	0.95 (0.30 to 2.99)	0.08	0.935	55.6	0.046	R	1.38	0.240
	GG vs. GA + AA	1.07 (0.55 to 2.10)	0.21	0.834	88.0	0.000	R	1.39	0.238
	GA vs. AA	0.81 (0.43 to 1.54)	0.64	0.524	0.0	0.503	F	1.85	0.138
	GG vs. AA	1.00 (0.27 to 3.62)	0.01	0.994	65.0	0.014	R	1.28	0.2708
	G vs. A	1.12 (0.58 to 2.14)	0.34	0.734	89.6	0.000	R	1.58	0.190
IL-6 174G/C	GG + GC vs. CC	1.10 (0.73 to 1.64)	0.44	0.658	61.4	0.051	R	0.36	0.752
	GG vs. GC + CC	1.02 (0.81 to 1.27)	0.15	0.879	17.4	0.304	F	−0.98	0.432
	GC vs. CC	1.13 (0.73 to 1.77)	0.55	0.581	64.4	0.038	R	0.53	0.647
	GG vs. CC	1.04 (0.80 to 1.36)	0.29	0.771	9.4	0.346	F	−0.46	0.693
	G vs. C	1.03 (0.90 to 1.18)	0.49	0.623	44.3	0.145	F	−0.08	0.943

OR: odds ratio; CI: confidence interval; *P*_A_: *P* value for test of the association; *P*_Q_: *P* value for between-study heterogeneity; F: a fixed-effects model; R: a random-effects model.

**Figure 2:** **Forest plots of TNF-α gene polymorphisms and lung cancer risk in overall populations (contrast GG + GA vs. AA).** OR: odds ratio; TNF-α: tumor necrosis factor-alpha.

In order to explore the source of heterogeneity, meta-regression was performed for the dominant model of TNF-α-308G/A. As shown in Table 4, detection method (*P* = 0.485) and region (*P* = 0.121) were both not the factors influencing the pooled effect for the meta-analysis. Moreover, the subgroup analyses (Table 5) demonstrated that mutant gene G acted as a dominant gene (OR = 0.12, 95% CI: 0.03 to 0.54; *P* = 0.006).

**Table 4:** **Meta-regression for TNF-α polymorphisms and susceptibility to lung cancer (GG + GA vs. AA)**

	**Coefficient**	**Standard Error**	***t***	***P***	**95% CI**
Region	2.652	1.235	2.15	0.121	−1.278 to 6.582
Detection method	−0.741	0.933	−0.79	0.485	−3.710 to 2.229
Constant	−3.278	2.817	−1.16	0.329	−12.244 to 5.687

**Table 5:** **TNF-α polymorphisms (GG + GA vs. AA) and susceptibility to lung cancer by subgroup analyses of region and detection method**

		***N***	***I*** ^**2**^	***P*** **value for heterogeneity**	**OR (95% CI)**	***Z***	***P***
Region	Europe	5	12.2	0.336	1.40 (0.70 to 2.78)	0.95	0.342
	Asia	1			0.12 (0.03 to 0.54)	2.77	0.006
Detection method	Real-time PCR	1			1.27 (0.30 to 5.39)	0.33	0.743
	PCR-RFLP	4	54.5	0.086	0.60 (0.15 to 2.38)	0.73	0.465
	PCR-SSP	1			10.57 (0.58 to 192.90)	1.59	0.112

PCR: polymerase chain reaction; PCR-RFLP: polymerase chain reaction-restriction fragment length polymorphism; PCR-SSP: polymerase chain reaction-sequence specific primer; *N*: number of enrolled studies; OR: odds ratio; 95% CI: 95% confidence interval.

#### IL-6-174G/C and lung cancer susceptibility

Four case-control studies investigated the association between the IL-6-174G/C and lung cancer susceptibility, containing 719 cases and 1,252 controls. All the studies were carried out in Europe. Results for the five comparison models are listed in Table 3. Similarly, no significant differences were observed in all comparison models with high heterogeneity (*I*^2^ > 50%) across studies researching GG + GC vs. CC and GC vs. CC (dominant model, GG + GC vs. CC: OR = 1.10, 95% CI: 0.73 to 1.64, *P* = 0.658; recessive model, GG vs. GC + CC: OR = 1.02, 95% CI: 0.81 to 1.27, *P* = 0.879; heterozygous genotype comparison, GC vs. CC: OR = 1.13, 95% CI: 0.73 to 1.77, *P* = 0.581; homozygous genotype comparison, GG vs. CC: OR = 1.04, 95% CI: 0.80 to 1.36, *P* = 0.771; allele comparison, G vs. C: OR = 1.03, 95% CI: 0.90 to 1.18, *P* = 0.623). Forest plot for the dominant model of IL-6-174G/C is shown in Figure 3.

**Figure 3:** **Forest plots of IL-6 gene polymorphisms and lung cancer risk in overall populations (contrast GG + GC vs. CC).** IL-6: interleukin 6; OR: odds ratio.

#### Publication bias

According to Egger’s linear regression test, no publication bias existed in all of the comparisons for both loci (Table 3). Moreover, the shape of funnel plots also suggest no publication bias among the studies focusing on TNF-α or IL-6 gene polymorphisms and lung cancer risk (Figure 4).

**Figure 4:** **Funnel plots of the odds ratios of lung cancer for TNF-α and IL-6 polymorphisms by number of individual studies. (A)** TNF-α gene polymorphism; **(B)** IL-6 gene polymorphism. IL-6: interleukin 6; OR, odds ratio; TNF-α: tumor necrosis factor-alpha.

#### Sensitivity analysis

Sensitivity analysis was done for each result, and the pooled OR remained unchanged after removing the maximum-weight study, indicating high reliability in our conclusions (data not shown).

## Discussion

Although the relationship between TNF-α (-308G/A) or IL-6 (174G/C) polymorphisms and cancer susceptibility [19-21] has been investigated previously, no studies were performed to specifically explore their association with the risk of lung cancer using a meta-analysis method. The present meta-analysis included eight studies, involving 1,676 cases and 2,267 controls. The results indicated no significant lung cancer susceptibility with TNF-α-308G/A or IL-6-174G/C polymorphism in the overall study populations. Our findings are in accordance with most of the related studies summarized in this meta-analysis. Sensitivity and publication bias analyses ensured the reliability of the conclusions.

Theoretically, genetic polymorphisms in the promoter region of the TNF-α and IL-6 genes could modulate their protein expression. For example, the G to A transition in the promoter region at position -308 results in higher expression levels of TNF-α [10,22]. Homozygotes for the G allele have higher plasma IL-6 levels than carriers homozygous for the C allele [11,23]. However, the current evidence provides a negative outcome, which may be explained by the fact that a single polymorphism/gene might have a limited impact on lung cancer susceptibility. Our results do not exclude the possibility that other polymorphisms or haplotypes in the TNF-α and IL-6 gene could be related to lung carcinogenesis. For example, Liang *et al*. demonstrated that G-to-A alteration at the -238G locus of the TNF-α gene and C-to-G alteration at the -572C locus of the IL-6 gene correlated with the development of lung cancers [24]. Chen *et al*. showed that a two-single-nucleotide polymorphism (SNP) CC (-6331C and -572C) IL-6 promoter haplotype was significantly more common among cases than among controls in both groups, indicating this haplotype is associated with increased lung cancer risk [25]. Therefore, comprehensive haplotype-based or multiple SNP-based strategies may provide more precise information on the genetic contribution of TNF-α or IL-6 to cancer etiology in the future [21].

In addition, there were some limitations in this meta-analysis that we need to pay attention to. First, our results were based on unadjusted estimates and a relatively limited study number made it impossible to perform subgroup analysis stratified by ethnicity, smoking status, and different types of lung cancer. Some investigators pointed out that cancer risk was significantly increased for individuals with the CC genotype of IL-6 in African populations, but not in Caucasian populations [20]. The lack of the population of Africa may lead to the decrease of studies and cause a deviation to final result. As we know, lung cancer is broadly classified into two subtypes basing on the microscopic appearance of the tumor cells: small-cell lung cancer and non-small-cell lung cancer. Moreover, according to pathological pattern, lung cancer is classified into several subtypes, including squamous cell carcinoma, adenocarcinoma, and bronchioloalveolar carcinoma. They do not share the same pathogenesis, which may complicate the results. Maybe that is why Shih *et al*. [10] reached an opposite conclusion from Seifart *et al*. [12]. Second, lack of individual data of each study limited our precise estimation of the interactions between SNP-SNP or SNP-environment factors.

## Conclusions

In summary, the present meta-analysis demonstrates no significant association between TNF-α-308G/A or IL-6-174G/C and susceptibility to lung cancer. However, further study is needed to evaluate the effects of TNF-α or IL-6 polymorphisms on lung cancer susceptibility by using large-sample case-control studies and involving different ethnicity, smoking status, or pathological-type descriptions.
